The article "Intelligent Algorithm-Based Analysis on Ultrasound Image Characteristics of Patients with Lower Extremity Arteriosclerosis Occlusion and Its Correlation with Diabetic Mellitus Foot" was published in 2021. Journal: J Healthc Eng.

# Intelligent Algorithm-Based Analysis on Ultrasound Image Characteristics of Patients with Lower Extremity Arteriosclerosis Occlusion and Its Correlation with Diabetic Mellitus Foot

**DOI:** 10.1155/2021/7758206

**Published:** 2021-09-25

**Authors:** YunShuang Wu, Yan Shen, Hailing Sun

**Affiliations:** ^1^Department of Ultrasound, Nanjing Integrated Traditional Chinese and Western Medicine Hospital, Affiliated with Nanjing University of Chinese Medicine, Nanjing 210014, Jiangsu, China; ^2^Department of Ultrasound, Lianshui County People's Hospital, Lianshui, Huai'an 223400, Jiangsu, China; ^3^Department of Ultrasound, Hongze District People's Hospital, Huai'an 223100, Jiangsu, China

## Abstract

**Objective:**

The study focused on the correlation between lower extremity arteriosclerosis and diabetic mellitus (DM) foot, and it was explored by virtue of ultrasound images processed by an intelligent algorithm.

**Methods:**

A total of 60 DM foot patients admitted to our hospital in the past three years were selected and divided into two groups according to their condition. Patients with DM foot alone were in group B (30 cases), and patients with DM foot combined with lower extremity arteriosclerosis occlusion were in group C (30 cases). 30 healthy people were in group A as a control. Color Doppler ultrasound was used to examine the arteries of the lower extremities of all subjects. It the intramedia thickness (IMT) from the femoral artery to the dorsal foot artery was recorded, whether there was plaque in the artery or knowing the size of the plaque, its echo, and distribution, and whether the artery had stenosis. Next, the stenosis percentage was calculated. Additionally, the general information of patients was analyzed. At the same time, an intelligent algorithm was used to process ultrasound images, and its effects on image quality were evaluated.

**Results:**

Doppler ultrasound images processed by Artificial Bee Colony (ABC) had less noise and better quality, and key information about the lesion was clearly displayed. There was no statistical difference between the general data of the three groups of patients; group B and group C had higher IMT value, plaque incidence, arterial stenosis incidence, and degree of stenosis versus group A, and there were statistically significant differences between groups B and C. In particular, the incidence of femoral artery stenosis and the degree of stenosis were significantly higher in group C than in group B. The rate of stenosis above grade I in group C was as high as 71%, while that in group B was only 19%; in Group C, the incidence of stenosis above grade II was 30%, and that in group B was 13.1%. Compared with group A, group B and group C had decreased peak arterial blood velocity (PSV), resistance index (RI), and pulse index (PI), and there were statistically significant differences between groups B and C.

**Conclusion:**

DM foot is a risk factor for arteriosclerosis occlusion; color Doppler ultrasound demonstrates good diagnostic effects on arteriosclerosis occlusion; the algorithm proposed in this study can improve the quality of Doppler ultrasound images and has a high application value.

## 1. Introduction

In recent years, with the continuous improvement of people's living standards and changes in dietary structure, the incidence of diabetes mellitus (DM) foot has been increasing year by year [1]. It is the third most common disease after tumors and cardiovascular diseases. DM foot is a common complication of DM patients. Statistics show that 15% of DM patients worldwide have foot ulcers and gangrene [2]. 50% of patients with amputation each year are DM patients, and more than 85% of these patients are amputated because of worsening foot ulcers leading to deep infection or gangrene. Domestic clinical data show that DM foot patients account for 2% of outpatients and 8% to 12% of inpatients. The per capita treatment cost for DM foot is more than 10,000 yuan. Worldwide, the incidence of DM foot is high, and the prognosis is poor [3].

As for why DM patients develop DM foot, it may be related to the influence of DM on the cardiac and cerebral vessels. To some extent, DM can be regarded as a cardiovascular and cerebrovascular disease and affects almost every blood vessel. The abnormal metabolism caused by DM can lead to changes in the structure and functions of arteries. These changes occur even before DM is diagnosed [4]. Peripheral arterial disease (PAD) is common in DM patients. It is a lower extremity occlusive disease, and its clinical symptoms are not obvious. PAD is an important indicator of thrombotic diseases of arteriosclerosis [5]. Statistics reveal that more than 40% of PAD patients suffer from DM, and DM is the strongest threat factor for PAD. Unlike PAD caused by other factors, DM is closely related to femoral-popliteal PAD and tibial artery PAD (below the knee). The DM foot arises from lower limb ischemia caused by arteriosclerosis occlusion [6]. Above, there is a huge correlation between DM foot and lower extremity arteriosclerosis occlusion. There are many commonalities but are different. Research has found that patients with both PAD and DM foot have a more complicated condition than patients with one of them alone, and the probability of cardiovascular diseases is greatly increased [7]. At present, the relationship between the two remains unclear. In the study, the correlation between the two was explored, in order to provide reference and basis for clinical research.

At present, the methods to diagnose lower extremity arteriosclerosis occlusion mainly include digital subtraction angiography (DSA), magnetic resonance angiography (MRA), CT angiography (CTA), and Doppler ultrasound. Among them, DSA is the recognized gold standard for peripheral vascular examination, but it is often not easily accepted by patients because it is invasive and expensive. As ultrasound technology marches forward continuously, it has been widely used in the detection of vascular diseases, especially in the research of atherosclerosis, because of its advantages, such as noninvasive, fast, efficient, safe, and accurate [8]. Statistics show that the accuracy of ultrasound examination for intraplaque hemorrhage is 90% and the sensitivity is 96%. B-mode ultrasound can display the anatomical images of the artery at longitudinal axis and at the transverse axis, providing rich information, such as artery thickness, plaque shape, size, range, and lumen stenosis and occlusion. Color blood flow imaging can reflect the blood filling and distribution state, which is of great significance for the evaluation of hemodynamic changes. In the early stage of atherosclerosis, it mainly manifests as expansion of the arterial wall or the thickening of MIT, which can be observed by ultrasound scan [9]. Thus, ultrasound has great advantages in the diagnosis of vascular diseases.

Nevertheless, its imaging effects are poor thanks to the reflection and random scattering. As a result, it is difficult to recognize the edges and details of the organs. Recently, Internet technology has developed rapidly, and some medical image processing technologies have also been developed, such as the arterial detection and tracking algorithm developed on the basis of ultrasound imaging, various ultrasonic 3D reconstruction algorithms, and computer-aided diagnostic systems. At present, the most widely used feature extraction and classification method in the field of medical image processing is the support vector machine. However, a large number of studies have shown that support vector machines are susceptible to extreme values in data classification and training. Therefore, in this article, the Artificial Bee Colony (ABC) was used to perform noise reduction and feature extraction on the ultrasound images of diabetes and arteriosclerosis occlusion [10], aiming to provide a scientific basis for the diagnosis and treatment of related diseases.

## 2. Materials and Methods

### 2.1. Research Subjects

60 patients with DM foot and DM foot combined with lower extremity arteriosclerosis occlusion who were hospitalized in the hospital from March 2019 to June 2019 were selected as the research subjects. 30 healthy subjects were selected into group A as a control. The 30 subjects in group B were patients with DM foot alone. The diagnostic criteria of DM foot were based on the standards drawn up by the first DM foot academic conference of the Chinese Medical Association Diabetes Mellitus Society. The 30 subjects in group C were patients with DM foot and lower extremity arteriosclerosis occlusion. The diagnostic criteria for lower extremity arteriosclerosis occlusion were as follows. (1) Those with intermittent claudication; resting pain; soreness, swelling, numbness, and numbness (patients with one or more of them was included); dystrophic changes in skin, hair, muscles, and nails; and ulcers or gangrene were included. (2) The affected swelled and the pulsation of the middle artery was weakened or disappeared. (3) Those with sclerosis changes on fundus examination; electrocardiogram showing coronary artery ischemia, left ventricular hypertrophy, or old myocardial infarction; and Doppler or angiography showing limb arteriosclerosis were also included. The subjects were 62 × 6.5 years old on average, including 44 males and 46 females. All subjects need to be free of coronary heart disease, hyperlipidemia, and other cardiovascular and cerebrovascular diseases, with no long-term smoking history. The study met the requirements of medical ethics and the patients had signed an inform consent form.

### 2.2. Examination Methods

#### 2.2.1. Inspection Instrument

Philips iu22 color Doppler ultrasonic diagnostic instrument, with a linear array probe, the probe frequency is 2–9 MHz. During the inspection process, conditions, such as emission energy, total gain, contrast, time gain compensation, and lateral gain compensation, need to be kept basically unchanged.

#### 2.2.2. Inspection Content

The patient stayed in the supine and prone positions, and two-dimensional ultrasound scan was performed on the femoral artery, popliteal artery, anterior tibial artery, posterior tibial artery, dorsal foot artery lumen, and inner membrane of both lower limbs. The lumen inner diameter and intramedia thickness (IMT) were measured. It was observed that there were plaques on the tube wall, the position of plaques, and that there was stenosis in the lumen. The stenosis percentage was then calculated. Color Doppler was used to observe the blood vessel filling, and spectrum Doppler was used to detect blood flow spectrum. After a clear spectrum appeared, the blood flow parameters PSV, RI, and PI were measured. During the inspection, it should be noted not to compress the artery too much, and the angle between the sound beam and the blood flow direction should be less than 60°; each index is measured 3 times, and the average value is taken.

### 2.3. Image Processing

A total of 220 ultrasound images are collected as research data. Then, the NL algorithm is used to reduce the noise of the image. The original noise image is *Y* ∈ *R*^*M*×*N*^, and the image NL(*Y*) after noise reduction was

(1) $$\begin{array}{c} \text{NL}\left(Y\left(p\right)\right)=\sum_{q=1}^{M\times N}w\left(p,q\right)=1, \end{array}$$

where *p* are the pixels to be denoised and *q* are the other pixels. *w*(*p*, *q*) is the weight, 0 ≤ *w*(*p*, *q*) ≤ 1, and ∑_*q*=1_^*M*×*N*^*w*(*p*, *q*)=1. The calculation of *w*(*p*, *q*) is as follows:

(2) $$\begin{array}{c} w\left(p,q\right)=\frac{1}{Z\left(p\right)}\exp\left(-\frac{d\left(p,q\right)}{h^{2}}\right). \end{array}$$

Then, the weighted Gaussian distance is used to judge the similarity:

(3) $$\begin{array}{c} d\left(p,q\right)=G_{p}{\left\|g\left(N_{p}\right)-g\left(N_{q}\right)\right\|}^{2}, \end{array}$$

where *G*_*p*_ is the Gaussian weighting function and *Z*(*p*) is the normalization parameter:

(4) $$\begin{array}{c} Z\left(p\right)=\sum_{q=1}^{M\times N}\exp\left(-\frac{d\left(p,q\right)}{h^{2}}\right), \end{array}$$

where *h* are the attenuation control parameters. This algorithm has good noise reduction effects but long calculation time. In order to reduce the amount of calculation and shorten the calculation time, the search range is controlled in the large search box of (2 × *R*_search_+1) × (2 × *R*_search_+1).

#### 2.3.1. Feature Extraction

The ultrasonic image features are divided into basic texture features and gray-level cooccurrence matrix features. The gray mean value of the *k* subblock is defined as

(5) $$\begin{array}{c} {\bar{y}}_{k}=\frac{1}{L2}\sum_{i=1}^{L}\sum_{j=1}^{L}{\left[y_{k}\left(i,j\right)-{\bar{y}}_{k}\right]}^{2}. \end{array}$$

The gray-level variance *σ*^2^(*y*_*k*_) of the *k* subblock is defined as follows:

(6) $$\begin{array}{c} \sigma^{2}\left(y_{k}\right)=\frac{1}{L2}\sum_{i=1}^{L}\sum_{j=1}^{L}{\left[y_{k}\left(i,j\right)-{\bar{y}}_{k}\right]}^{2}. \end{array}$$

The probability that the pixels (*i*′, *j*′) with distance *d*, angle *θ*, and gray value *g*_2_ appear at the same time is as follows:

(7) $$\begin{array}{c} P_{\theta ,d}\left(g_{{}_{1}},g_{{}_{2}}\right)=\#\left\{\left(i,j\right),\left(i^{\prime },j^{\prime }\right)\in M\times N|f\left(i,j\right)=g_{1},f\left(i^{\prime },j^{\prime }\right)=g_{2}\right\}, \end{array}$$

where #{·} represents the number of elements in the set. For the sake of simplicity, *θ* and *d* are ignored, and the matrix is normalized as follows:

(8) $$\begin{array}{c} \frac{P_{\theta ,d}\left(g_{1},g_{2}\right)}{R}⟶P\left(g_{1},g_{2}\right), \end{array}$$

where *R* is the normalization constant and its value is the total number of point pairs in the gray-level cooccurrence matrix. CON is the contrast, and it can reflect the clarity and texture of the image. A greater grayscale difference of the pixel pair value leads to a greater value of CON:

(9) $$\begin{array}{c} \text{CON}=\sum_{g_{1}=0}^{N_{g}-1}\sum_{g_{2}=0}^{N_{g}-1}{\left|g_{1}-g_{2}\right|}^{2}p^{2}\left(g_{1}-g_{2}\right). \end{array}$$

Entropy ENT can be a measure of the complexity of the image texture, and it is calculated as follows:

(10) $$\begin{array}{c} \text{ENT}=-\sum_{g_{1}=0}^{N_{g}-1}\sum_{g_{2}=0}^{N_{g}-1}P\left(g_{1},g_{2}\right)\log\left[P\left(g_{1},g_{2}\right)\right]. \end{array}$$

The linear dependence of the image gray level depends on COR:

(11) $$\begin{array}{c} \text{COR}=\frac{\sum_{g_{1}=0}^{N_{g}-1}\sum_{g_{2}=0}^{N_{g}-1}g_{1}g_{2}P\left(g_{1},g_{2}\right)-\mu_{g_{1}}\mu_{g_{2}}}{\sigma_{g_{1}}\sigma_{g_{2}}}. \end{array}$$

Energy ENG can reflect the uniformity of the image gray distribution and the thickness of the texture:

(12) $$\begin{array}{c} \text{ENG}=-\sum_{g_{1}=0}^{N_{g}-1}\sum_{g_{2}=0}^{N_{g}-1}p^{2}\left(g_{1},g_{2}\right). \end{array}$$

### 2.4. Observation Indicators

The measurement of intramedia thickness (IMT) takes the average value of the left and right sides, and the thickest part of the arterial wall is measured in the diastolic phase of each segment of the lower limbs. It should be noted to be away from the plaque position during the measurement. IMT ≤ 0.9 mm is the normal value, and IMT > 0.9 mm is the thickened IMT. Plaque is defined as: localized thickening of blood vessel wall greater than 1.2 mm or diffuse thickening of blood vessel greater than 1.2 mm. The calculation of vascular stenosis rate depends on the percentage reduction of inner diameter: vascular stenosis rate = ((*d*_2_ − *d*_1_)/*d*_2_) × 100% (*d*_1_ is the inner diameter of the lumen at the stenosis and *d*_2_ is the original inner diameter of the lumen). The grades of stenosis were as follows: grade 0, no stenosis; grade I, stenosis rate 1%∼19%; grade II, stenosis 20%∼49%; grade III, stenosis 50%∼99%; grade IV, occlusion, no blood flow information. If there are multiple plaques or stenosis in the same segment of blood vessel, the most severe part of the stenosis shall prevail.

### 2.5. Statistics

The data was processed by SPSS 17.0 software. The measurement data were expressed as $\left(\bar{x}\pm s\right)$. The comparison of data between groups adopted analysis of variance, and the *x*^2^ test was used to test the count data. *P* < 0.05 was the threshold for significance.

## 3. Results

### 3.1. The Basic Information of Subjects

The basic information of the subjects was shown in Table 1. The average ages of A, B, and C groups were 65.1 ± 6.8, 66.2 ± 5.4, and 64.2 ± 5.9, respectively. The number of male subjects in the three groups was 16, 18, and 17, respectively, and the number of female subjects was 14, 12, and 13, respectively; the proportions of smokers in each group were 16%, 15.1%, and 15.3%. It was noted that there was no significant difference between the general data of the three groups of subjects and it was comparable.

### 3.2. Ultrasound Images and Processing Results

The original ultrasound image and the processed image were shown in Figure 1. From column A in Figure 1, it was noted that although Doppler color ultrasound can reflect the arterial thickness, plaque shape, size, range, luminal stenosis and occlusion, blood flow filling, and other information in a comprehensive and detailed manner, the figure had much noise, with poor clarity and quality. It failed to show the edge and detailed information of diseased parts and tissue. As for column B in Figure 1, the clarity of the image was improved a lot, and the noise has also been reduced. At the same time, the key information of the disease was extracted, and the redundant information was removed that had nothing to do with the disease, to highlight the focus of the disease.

### 3.3. The Intramedia Thickness and Hemodynamic Test Results of the Lower Extremity Arteries of Each Group

The IMT measurement results of both lower limbs in the three groups were shown in Figure 2. Compared with group A, subjects in groups B and C had thicker IMT in the lower limb femoral artery, popliteal artery, anterior tibial artery, posterior tibial artery, and dorsal foot artery, and the difference was statistically significant, *P* < 0.05. The thickening of IMT in group C was more obvious versus group B, and the difference was statistically significant, *P* < 0.05.

The hemodynamic results of each group were shown in Figure 3. The test indicators included peak systolic velocity (PSV), resistance index (RI), and pulse index (PI), and the detection was located in femoral artery, popliteal artery, anterior tibial artery, posterior tibial artery, and dorsal foot artery. Compared with group A, PSV, RI, and PI of groups B and C decreased, and the difference was statistically significant, *P* < 0.05, and the decrease in group B was more obvious versus group C, and the difference was statistically significant, *P* < 0.05.

### 3.4. Occurrence and Distribution of Atherosclerotic Plaques in the Lower Extremities of Each Group

Two-dimensional ultrasound results showed that the intima surface of the lower extremity arteries in groups B and C were not smooth, and there were patches or dots with localized or diffuse distribution and uneven echo. The plaques at the femoral artery were mostly single and large in volume. The plaques were often found at the bifurcation. The plaques of the popliteal artery, anterior tibial, posterior tibial, and dorsal foot artery were mostly diffusely distributed dots echoes and small in volume.  Figure 4 showed the plaque incidence in each group, where (a) was the total number of arteries, (b) was the number of plaque arteries in each arterial segment, and (c) was the probability of plaque in each arterial segment. Compared with A, the incidence of plaque in the lower limb femoral artery, popliteal artery, anterior tibial artery, posterior tibial artery, and dorsal foot artery in the groups B and C was higher, *P* < 0.05, and the difference was statistically significant. The incidence of arterial plaque in each segment of the C group was higher than that of the B group, and the difference was statistically significant, *P* < 0.05.

### 3.5. Occurrence of Arteriosclerosis and Stenosis of the Lower Extremities

Two-dimensional ultrasound results showed that the arterial intima of the lower extremities of the two groups B and C showed varying degrees of thickening and plaques of different sizes and irregular shapes protruding into the lumen, resulting in varying degrees of stenosis of the vascular lumen. Figures 5–9 showed the occurrence and distribution of stenosis in each group. Compared with group A, the lower extremity arterial stenosis rate of groups B and C was higher, and the difference was statistically significant, *P* < 0.05. The incidence of stenosis in of group C was higher than that of group B, and the difference was statistically significant, *P* < 0.05. In particular, the incidence of femoral artery stenosis and the degree of stenosis was higher in group C than in group B. The stenosis rate of grade I and above in group C was as high as 71%, while that in group B was only 19%; in group C, the stenosis rate of grade II and above was 30%, and that in group B was 13.1%.

## 4. Discussion

In China, diabetes is a common disease that threatens the lives and health of people. With the development of economy and the gradual westernization of lifestyle, the incidence of diabetes continues to rise [11]. DM foot is one of the most common complications of diabetes [12]. Studies have shown that 15 out of every 100 diabetic patients will suffer from DM foot. Clinical data show that diabetes is the culprit of 50% of amputation patients every year. In general, DM foot can be divided into two types. One is DM foot combined with lower extremity arteriosclerosis occlusion, with the lower extremity arteriosclerosis being the main pathological change. It manifests as the coldness of the lower extremities, numbness, poor skin nutrition, and weakened or disappeared artery pulsation in distant end of lower extremities, that is, ischemic diabetes [13]. The other is DM foot with no obvious arteriosclerosis of the lower extremities, that is, nonischemic diabetes. Such patients have no obvious symptoms of lower limb ischemia, and the pulsation of dorsal foot artery and posterior tibial artery is also good. Clinical statistics show that the proportion of DM foot combined with lower extremity arteriosclerosis occlusion is different among countries, regions, and races [14]. The reason may be that we have different definitions of the two diseases, which has caused ambiguity. The international definitions of DM foot and fine arteriosclerosis occlusion are as follows. DM foot refers to the foot ischemia, infection, or neuropathy in diabetic patients; lower extremity arteriosclerosis occlusion is a systemic arterial disease, and it manifests as the appearance of atherosclerotic plaque, degeneration or calcification of the middle layer of the tissue, and the formation of secondary thrombosis in the lumen, which will eventually narrow or even completely occlude the lumen. In severe cases, ischemia in lower extremities may cause acronecrosis [15]. As per the definition, both DM foot and lower extremity arterial occlusion are related to ischemia. When a diabetic person has lower extremity arterial bleeding, whether it should be diagnosed as diabetic foot or lower extremity arteriosclerosis occlusion is a common problem that currently plagues clinicians [16]. If diagnosed as DM foot, it will enlarge the influence of DM foot and reduce the detection rate of arteriosclerosis occlusion; if diagnosed as lower extremity arteriosclerosis occlusion, it will reduce the detection rate of DM foot combined with lower extremity arteriosclerosis occlusion [17]. For the relationship between the two, scholars have used mathematical sets to express it; that is, those with DM foot alone and those with lower extremity arteriosclerosis occlusion alone are in mutually independent subsets, and those in the intersection have DM foot combined with arteriosclerosis occlusion. Hence, it is important to explore the difference and connection between the two [18].

Currently, except for the diagnosis method based on the clinical systems, the main methods to diagnose DM foot and lower extremity arteriosclerosis occlusion include DSA, MRA, CTA, and Doppler ultrasound. Among them, DSA is the gold standard for peripheral blood vessel examination, but it is invasive and expensive and thus poorly accepted by patients. Ultrasound examination has been widely used in clinical vascular examinations, especially the diagnosis of atherosclerosis, because of its fast speed, noninvasiveness, accuracy, and simple operation. It can detect early atherosclerosis and the location of small nonstenotic atherosclerotic plaques. Despite many advantages, the ultrasound examination is affected by reflection and random scattering, the image has large noise, and the edge of the lesion is often blurred. To further improve the quality of ultrasound images to more accurately grasp the patient's disease information, researchers have applied various image processing techniques to ultrasound image processing, such as the arterial detection and tracking algorithm developed on the basis of ultrasound images [19]. In this study, the ABC algorithm was used to process the Doppler ultrasound images of all subjects. The study found that compared with the original image, the processed image was clearer, and the lesion features were more prominent. Then, the relationship between DM foot and lower extremity arteriosclerosis occlusion was analyzed on the basis. The study found that patients with DM foot combined with lower extremity arteriosclerosis occlusion had a higher incidence of lower extremity plaque and severe vascular stenosis compared with patients with DM foot alone. This suggested that DM foot is a risk factor for lower extremity arteriosclerosis occlusion.

## 5. Conclusion

In this study, patients with DM foot combined with PDA were selected, and they were analyzed for lower extremity arterial stenosis and plaque occurrence, as well as MIT thickness. Then, the correlation between DM foot and lower extremity arteriosclerosis occlusion was explored. It was found that DM foot was one of the risk factors for lower extremity arteriosclerosis occlusion, which negatively affect the prognosis of extremity arteriosclerosis occlusion. Meanwhile, an intelligent algorithm was used to process Doppler ultrasound images. It was found that the algorithm can highlight lesion information and improve image quality, with high application value and prospects. However, some limitations in the study should be noted. The sample size is small, which will reduce the power of the study. In the follow-up, an expanded sample size is necessary to strengthen the findings of the study.

## Figures and Tables

**Figure 1:** Comparison of the original ultrasound image and the processed image. *Note*. (a) The original image and (b) the processed image.

**Figure 2:** Comparison of intramedia thickness results of each group. *Note*. Compared with group A, ^*∗*^*P* < 0.05; compared with group B, ^#^*P* < 0.05.

**Figure 3:** Hemodynamic examination results of each group. *Note*. Compared with group A, ^*∗*^*P* < 0.05; compared with group B, ^#^*P* < 0.05. (a) Femoral artery. (b) Popliteal artery. (c) Tibial artery before. (d) Posterior tibial artery. (e) Dorsalis pedis artery.

**Figure 4:** The occurrence and distribution of atherosclerotic plaques in the lower extremities of each group. *Note*. Compared with group A, ^*∗*^*P* < 0.05; compared with group B, ^#^*P* < 0.05.

**Figure 5:** The occurrence of femoral artery stenosis in each group. (a) Total number of arteries in each group. (b) The number of arteries with stenosis in each group. (c) The occurrence probability of arterial stenosis in each group.

**Figure 6:** The occurrence of popliteal artery stenosis in each group. (a) Total number of arteries in each group. (b) The number of arteries with stenosis in each group. (c) The occurrence probability of arterial stenosis in each group.

**Figure 7:** The occurrence of anterior tibial artery stenosis in each group. (a) Total number of arteries in each group. (b) The number of arteries with stenosis in each group. (c) The occurrence probability of arterial stenosis in each group.

**Figure 8:** Occurrence of posterior tibial artery stenosis in each group. (a) Total number of arteries in each group. (b) The number of arteries with stenosis in each group. (c) The occurrence probability of arterial stenosis in each group.

**Figure 9:** Occurrence of dorsal artery stenosis in each group. (a) Total number of arteries in each group. (b) The number of arteries with stenosis in each group. (c) The occurrence probability of arterial stenosis in each group.

**Table 1:** The basic information of subjects.

Item		A (30 cases)	B (30 cases)	C (30 cases)
Case		30	30	30
Age (year)		65.1 ± 6.8	66.2 ± 5.4	64.2 ± 5.9
Gender	Male	16	18	17
	Female	14	12	13
Proportion of smokers (%)		16	15.1	15.3
TC (mol/L)		4.66 ± 1.08	4.55 ± 1.13	4.61 ± 1.14
TG (mol/L)		2.06 ± 1.16	2.08 ± 1.12	4.07 ± 1.19

## Data Availability

The data used to support the findings of this study are available from the corresponding author upon request.
